# The Effect of Toothpastes Containing Natural Ingredients Such As Theobromine and Caffeine on Enamel Microhardness: An In Vitro Study

**DOI:** 10.1155/2021/3304543

**Published:** 2021-10-22

**Authors:** Farzaneh Golfeshan, Seyed Ali Mosaddad, Faezeh Ghaderi

**Affiliations:** ^1^Orthodontics Research Center, Department of Orthodontics, School of Dentistry, Shiraz University of Medical Sciences, Shiraz, Iran; ^2^Student Research Committee, Shiraz University of Medical Sciences, Shiraz, Iran; ^3^Oral and Dental Disease Research Center, Department of Pediatric Dentistry, School of Dentistry, Shiraz University of Medical Sciences, Shiraz, Iran

## Abstract

The current study aimed to investigate the effect of biocompatible kinds of toothpastes containing natural ingredients such as theobromine and caffeine on the enamel microhardness after demineralization. 72 maxillary premolar teeth extracted for orthodontic purposes were used in this study. Primary enamel surface microhardness examinations were performed using a Digital Micro Vickers Hardness Tester following the Knoop technique (50 g load for 15 s with three indentations at various points). The specimens were immersed in lactic acid (pH = 5.4) for 7 days, washed with distilled water, dried, and then retested for microhardness. According to the type of toothpaste used for brushing, all specimens were categorized as follows: Group 1, Theodent classic® toothpaste (theobromine); Group 2, Power Energy toothpaste (caffeine); Group 3, Colgate toothpaste (fluoride); and Group 4, distilled water as the negative control. The specimens were retested for enamel microhardness after brushing 2 times a day for one month. After brushing with different types of toothpaste, for all experiment groups, the increase in microhardness values in the demineralized enamel surfaces was significant and there were significant differences between them (*p* value <0.05). The fluoride group had the highest microhardness and had a significant difference with the caffeine and distilled water groups, but there was no significant difference with the theobromine group (*p* value <0.05). In the theobromine group, the hardness was considerably higher than in the caffeine and distilled water groups. There was no significant difference between the caffeine and distilled water groups. Theobromine toothpaste had the same remineralization effect as that of fluoride toothpaste, while caffeine toothpaste had no positive effect on the remineralization process.

## 1. Introduction

The enamel has natural demineralization and remineralization cycles; enhanced demineralization of the tooth surface causes dental caries, which in turn results in continual mineral loss from the crown or root of teeth. This process is mainly caused by bacteria. There are five factors that can stimulate the occurrence of caries, including accumulation of plaques, high consumption of carbohydrate or acidic foods and beverages, natural ingredients like saliva and pellicle, and fluoride levels. It is worth noting that the first three factors are mentioned as the main causes of caries [1].

Scholars have been reporting on enamel remineralization for about one century, and it is noted that “the noninvasive treatment of early caries lesions by remineralization has the potential to be the major advance in the clinical management of the disease” [2]. Several techniques have been introduced to enhance the mechanical characteristics of enamel to avoid the early development of caries [3]. The most successful caries-preventive agent is fluoride [4]. High consumption of fluoride may result in fluorosis, damage to the teeth, dark stripes on teeth, and tooth loss. In addition, it may result in decreased intelligence in children who receive low levels of fluoride as well as early aging, abortion, and brittle bones [5]. It has been reported that fluoride consumption at a level more than 5 mg F/kg body weight for children and adults could cause acute toxic effects, while the lethal dose for children is considered to be 16 mg F/kg body weight and it is 32 mg F/kg body weight for adults [6]. Due to the side effects of these chemical components, an increasing public interest in natural or herbal-based healthcare products, especially in different kinds of toothpaste, is being observed. This incline is not only observed in cosmetic markets and dental practices but also in the scientific world [7]. An increasing amount of clinical study is being performed to verify the effectiveness of these products; thus, in terms of dental hygiene products, attention nowadays is paid to some natural and biocompatible alternatives to fluoride, like theobromine [4]. Theobromine (3, 7-dimethylxanthine) is a primary alkaloid derived from the *Theobroma cacao* plant [8]. It can also be found in cacao leaves, although its concentration is significantly lower [3]. Theobromine is a water-soluble, crystalline, bitter powder that is available in chocolates along with tea and other foods [8]. It is differentiated from caffeine by only one methyl group [9]. The molecular formula for theobromine is C_7_H_8_N_4_O_2_ [4]. It is proven that theobromine compounds can improve the hardness of the tooth enamel surface through stimulating interstitial reactions between the HA crystals and theobromine on the enamel surface [3]. Recently developed kinds of toothpaste contain theobromine can trigger remineralization without causing any toxicity.

All around the world, coffee is served, mainly because of its taste and its effect on both mental and physical activities. Mixed messages from scientists about the advantages or disadvantages of coffee are almost a weekly event [10]. Caffeine (1, 3, 7-trimethylxanthine) is a bitter, white crystalline purine, a methylxanthine alkaloid. In addition, chemically, it belongs to the adenine and guanine bases of deoxyribonucleic acid (DNA) and ribonucleic acid (RNA) [11]. *Coffea canephora* is rich in polyphenols, which are mentioned as potential agents that can prevent oral diseases, especially those related to biofilms. According to Cowan, the potential reasons for phenolic toxicity to microorganisms are enzymatic inhibition by oxidized compounds, possibly through reactions with sulfhydryl groups or nonspecific interactions with proteins [12]. Of all the documented bioactivities of coffee, a few show antioxidant, anticarcinogenic, and antimutagenic activities [13]. Different compounds are reported as the cause of the chemoprotective effects of coffee, which are mainly polyphenols, such as chlorogenic acids and their degradation products, as well as caffeine, kahweol, cafestol, and other phenolics [13]. Coffee can influence *Streptococcus mutans*, the organism that causes the development of dental caries. In addition, it is reported that roasted coffee has antiadhesive characteristics. Hence, it can intervene in the adhesion of *S. mutans* and the rest of the detrimental compounds to the teeth. Those who drink coffee regularly not only have caries-free teeth, but also their teeth are whiter as compared to others [10]. Because of this proven effect, nowadays, manufacturers produce toothpaste containing caffeine to utilize its antibacterial and mental-stimulating effect. Since there have always been conflicting reports in the field of dentistry about the effect of caffeine on dental health and no study has been done on the effect of caffeine-containing toothpaste on tooth enamel, we designed this study. In the present study, the effect of different kinds of toothpaste containing theobromine, caffeine, and fluoride on enamel microhardness was evaluated after artificial demineralization.

## 2. Materials and Methods

### 2.1. Teeth Preparation

72 maxillary premolar teeth with caries-free buccal surfaces that were extracted for orthodontic purposes were used in this study which was approved by the Ethical Committee of Shiraz University of Medical Sciences, Dental School with number 21804-37-01-98.

Then, all the teeth were rinsed with water and maintained in 70% ethanol until the experiment day. The teeth were mounted in a polyester mold (Figure 1). All the teeth were cleaned with a brush and pumice and stored in artificial saliva.

### 2.2. Enamel Microhardness Analysis

Primary enamel surface microhardness analyses were performed using a Digital Micro Vickers Hardness Tester machine following the Knoop technique (50 g load for 15 s with three indentations at various points) (SCTMC, model: MHV-1000Z, China). This machine can directly show the test mode, test force, indentation length, dwell time, test numbers, conversion scale, and date and time. It can use an optional Knoop indenter to measure Knoop hardness.

### 2.3. Demineralization Process

A solution of lactic acid (titration min. 90.0%) with pH 5.4 was used to demineralize the enamel surfaces. The specimens were immersed in the demineralized solution for 7 days, washed with distilled water, dried, and then retested for microhardness.

### 2.4. Application of Toothpastes

The samples were randomly categorized into four groups according to the type of toothpaste: Group 1, brushed with Theodent classic® toothpaste (Theodent classic™, Rennou, UK-853069003006); Group 2, brushed with Power Energy toothpaste (Power Energy, Denver, USA-86095200020); Group 3 (positive control) brushed with Colgate toothpaste (Colgate Regular and Colgate-Palmolive, Thailand); and Group 4 (negative control) treatment with distilled water. These kinds of toothpaste were chosen based on their similar excipients to exclude the effects of any dissimilar excipient and to only evaluate the effective component of each toothpaste.

The specimens were brushed twice a day for 1 month, and each brushing period lasted for 1 minute [1]; then, they were immersed in a solution containing toothpaste for 2 minutes. The quantity of toothpaste added to the solution was managed at a ratio of 1 : 33, where 3 g of paste was added to 10 mL of distilled water. The samples were retested for enamel microhardness after treatment with different kinds of toothpaste using the same method as the previous steps.

### 2.5. Statistical Analysis

Data analyses were administered using SPSS version 22. The normality of the data was evaluated using the Shapiro–Wilk test. In addition, the Wilcoxon signed-ranks test was used to evaluate differences in microhardness values between the initial, demineralization, and remineralization steps in each group. Differences in mean values between the experimental groups were investigated by the Kruskal–Wallis and Mann–Whitney tests.

## 3. Results

According to the results of the Shapiro–Wilk test, data were not distributed normally (*p* > 0.05); hence, nonparametric tests (i.e., Kruskal–Wallis and Mann–Whitney tests) were used to investigate differences in mean values of hardness between the study groups following the demineralization process and treatment.

### 3.1. Enamel Microhardness in Initial and Demineralization Phase

Table 1 presents the mean values of microhardness of four experimental groups in the initial (T1) and demineralization (T2) phases and the differences between these two steps (T1-T2). Microhardness values were significantly decreased after the demineralization process in each treatment group with no statistically significant differences between them.

### 3.2. Enamel Microhardness after Brushing

According to Table 2, a considerable increase in microhardness values (*p* < 0.05) after brushing could be seen in all groups. A significant difference was found in mean values between the four groups (*p* < 0.05).

### 3.3. Comparison of Microhardness Values

A post hoc analysis was done using a Mann–Whitney test, which revealed no significant difference between the fluoride and theobromine groups, while the microhardness values were significantly higher in these groups than in the caffeine and distilled water groups. The caffeine and distilled water groups had no statistically significant differences in their microhardness values (Table 3).

## 4. Discussion

In recent years, many studies have investigated the impact of early noninvasive treatment of incipient lesions through remineralization of the enamel surface [2]. As a result, some novel enamel remineralization systems have been introduced, some of which are currently being used in the clinical setting [14]. The primary method recommended to either prevent or reverse initial lesions is to use different kinds of toothpaste, followed by mouthwashes and gels with good active biocompounds. Active compounds as well as other necessary components are present in different kinds of toothpaste. Different active compounds that contribute to the promotion of enamel remineralization are present in different kinds of toothpaste, the most common compound being fluoride [15]. To prevent the side effects of fluoride, studies have been conducted to find a natural and biocompatible alternative to fluoride. According to various studies, theobromine is a good alternative to fluoride [15]. In this study, changes in enamel microhardness after demineralization followed by treatment with toothpaste containing theobromine, caffeine, and fluoride were investigated. After exposure to different kinds of toothpaste, the increase in microhardness values in the demineralized enamel surfaces of all four experimental groups were significant, and there were significant differences between their values (*p* value <0.05). The findings revealed no significant difference between the fluoride and theobromine groups, while the microhardness values were significantly higher in these groups than in the caffeine and distilled water groups. The caffeine and distilled water groups had no statistically significant differences in their microhardness values. The ability of fluoride to remineralize caries is the gold standard against which other remineralization systems must compete, either alone or in combination with fluoride. Currently, several acidulated fluoride products are available. The most common product is mouth rinse of sodium fluoride with phosphoric acid at pH 3.0–4.0, gels, and foams [16]. In the present study, the fluoride group had the highest hardness and had a significant difference with the caffeine and distilled water groups, but there was no significant difference with the theobromine group. In an in vitro study conducted by Sulistianingsih et al., fluoride (solution of 1000 ppm fluoride for 15 minutes) could increase the harness of enamel samples after artificial demineralization [17]. Arnold et al. demineralized the enamel surface of 90 human premolars in a hydroxyethyl cellulose solution at pH 4.8, followed by immersion of teeth in toothpaste slurry. They concluded that amine fluoride compounds in different kinds of toothpaste result in marked remineralization of caries like enamel lesions followed by sodium fluoride and sodium monofluorophosphate formulations [18]. The result of our study is the same as the previous studies in the literature about the remineralization effect of fluoride. The main components of hydroxyapatite in tooth enamel are phosphate ions (PO_4_^3–^) and calcium ions (Ca^2+^). There is a steady equilibrium among calcium and phosphate ions in saliva, in normal conditions, and in the crystalline hydroxyapatite that makes up 96% of tooth enamel. When pH is lower than the critical level (5.5 and 6.2 for enamel and dentin, respectively), it stimulates demineralization, that is, the dissolution of tooth mineral (hydroxyapatite). However, in cases where the natural buffer capacity of saliva results in increased pH, it causes remineralization. In situations where fluoride exists in oral fluids (i.e., saliva), the remineralization process results in the formation of fluorapatite, not hydroxyapatite. Fluoride ions (F^–^) replace hydroxyl groups (OH–) in the formation of the apatite crystal lattice. In other words, fluoride stimulates further remineralization [19].

Recently, some studies have mentioned theobromine as an effective remineralizing agent and a potent alternative to fluorides [8]. Nakamoto et al. mentioned theobromine and fluoride as substances that can enhance apatite crystal size, which is related to enamel surface microhardness [20]. In the present study, the specimens brushed with theobromine showed an increase in microhardness values significantly. The results showed that there was no significant difference between fluoride and theobromine, while a significant difference exists between these two groups and the caffeine and distilled water groups. There are some conflicting reports in the literature regarding the remineralization effect of theobromine in comparison to fluoride. Nakamoto et al. in their study reported that theobromine and fluoride had the same remineralization effects [20]. The result of the Nasution et al. study showed that fluoride had a higher remineralization effect than theobromine [4], also Parvathy et al. indicated that theobromine had less remineralization potential in comparison to a dentifrice containing fluoride and with no significant difference between the two groups [8]. Pribadi et al. studies reported that the surface hardness of enamel following immersion in theobromine cacao rind extract seems to be significantly higher than in the fluoride group [3]. The tooth enamel surface hardness can be affected by the exchange of minerals on the surface of the enamel [21]. Amaechi et al. reported that theobromine can cause the growth of new enamel and stimulates calcium and phosphate growth from the saliva to integrate into a crystal unit that is larger (by 4-folds) than hydroxyapatite. The combination of mineral placement as new enamel growth may cause alternations in enamel hardness [22].

All around the world, coffee is widely served, mainly because of its taste and its effect on both mental and physical activities [23]. Conflicting results are reported regarding the advantages or disadvantages of coffee. According to the currently available evidence, it cannot be argued that drinking coffee either protects or damages the arteries, as it has several useful antioxidants, or may stimulate anything from cancer to bone loss [10]. In limited amounts, coffee makes teeth healthier and whiter. In addition, it has several other health benefits.

Moreover, apart from keeping one alert and awake, coffee contains several health benefits. Coffee is not only a morning jolt, as it has components called antioxidants, which are useful. In a study conducted several years ago in California, a professor of environmental toxicology reported that the amount of antioxidants available in freshly brewed coffee is equal to three oranges. Generally, antioxidants have several potential benefits, such as preventing cardiovascular diseases and liver and colon cancers (among different types of cancer), type 2 diabetes, and Parkinson's disease [10].

In dentistry, there are two opposite reports about the effect of caffeine on tooth enamel. On the one hand, scientists at two Italian universities conducted laboratory tests and reported that coffee molecules could intervene with the adhesion of *S. mutans* on tooth enamel. The first author, Gabriella Gazzani, a university professor at the Department of Druggist Chemistry of Pavia University, reported that all coffee solutions contain high antiadhesive characteristics, mainly because of naturally occurring as well as roasting-stimulated molecules. She and other scholars at the University of Ancona investigated sampled green and roasted *Arabica* and *Robusta* coffee collected from various countries. They reported that all analyzed samples could prevent *S. mutans* adsorption and revealed inhibitory properties, ranging from 40.5 to 98.1% [10]. Some of other studies reported that the acidity of caffeine may promote the demineralization of the enamel surface [12]. On the other hand, Falster et al. in their study reported the negative effect of consumption of caffeine during pregnancy on the enamel microhardness of newborns [24]. Because of caffeine's anti-*S. mutans* properties and emotional effects, nowadays some toothpaste manufacturers add caffeine as the main component. So far, we could not find a study to evaluate the effect of caffeinated kinds of toothpaste on enamel hardness; therefore, we designed this study.

Because there was no available toothpaste whose only active ingredient was caffeine, in this study, we used Power Energy toothpaste, whose active ingredients were caffeine and xylitol. The mechanism of action of xylitol has been studied in various research; different kinds of toothpaste that contain xylitol not only decrease the number of *S. mutans* colonies in saliva and the level of secreted saliva but can also increase the pH value. Increased flow of saliva with high levels of calcium and phosphate and shorter duration of low plaque pH may result in remineralization. The anticaries property of xylitol is mainly due to its impact on plaque and cariogenic microorganisms [25]. The presence of xylitol in the caffeinated toothpaste used for the experiment was the major limitation of our study because we could not differentiate the effects of caffeine and xylitol on enamel microhardness. In the present study, the microhardness was increased after brushing with caffeinated toothpaste, but this increase was the same as in distilled water groups. It could be concluded that the caffeine in toothpaste did not have the ability to demineralize nor it had a negative effect on enamel microhardness. Toothpaste containing xylitol and caffeine had the same effect as distilled water. In a study conducted by Tange et al., they concluded that xylitol itself had the same remineralization effects as that of fluoride [26], but in our study, we found that toothpaste containing xylitol and caffeine had a significantly lower remineralization effect than fluoride. One of the reasons for this difference might be the presence of caffeine. Caffeine might have reduced the remineralization effect of xylitol.

The present study demonstrated a significant increase in hardness values in the negative control group (group 4) following treatment with distilled water (*p* value <0.05). It is well proved that brushing can remove the demineralized soft enamel layer. In addition, it exposes the underlying hard enamel layer, which in turn results in increased hardness of the enamel [27].

The limitations of this study were the lack of toothpaste in which the only active ingredient was caffeine, and the presence of xylitol in the caffeinated toothpaste that was used for the experiment, because of which we could not differentiate the effects of caffeine and xylitol on enamel microhardness, laboratory study, and the impossibility of investigating the antibiotic properties of caffeine in the oral environment.

## 5. Conclusion

There was no significant difference between the fluoride and theobromine groups, while the microhardness values were significantly higher in these groups than in the caffeine and distilled water groups. Therefore, theobromine is a good alternative to fluoride to overcome the side effects of fluoride in high concentrations. The caffeine and distilled water groups had no statistically significant differences in their microhardness values.

## Figures and Tables

**Figure 1:** Mounting the specimens.

**Table 1:** Enamel microhardness in the initial and demineralization phases in each group.

Group	Hardness mean value ± SD (KHN)			*p* value
	Initial hardness ± SD	Demineralization hardness ± SD	Diff 1 ± SD	
1 (theobromine)	235.96 ± 87.09	151.09 ± 82.76	84.86 ± 47.49	0.001
2 (caffeine)	216.40 ± 66.75	151.20 ± 64.03	65.20 ± 58.74	0.001
3 (fluoride)	214.48 ± 64.14	146.29 ± 69.26	68.18 ± 37.42	0.001
4 (distilled water)	247.37 ± 65.44	149.98 ± 64.42	97.39 ± 64.52	0.001
	0.457	0.996	0.146	

Diff 1 = initial–demineralization; SD: standard deviation.

**Table 2:** Enamel microhardness values after brushing in each four groups.

Group	Hardness mean value ± SD (KHN)			*p* value
	Demineralization hardness ± SD	Remineralization hardness ± SD	Diff 2 ± SD	
1 (theobromine)	151.09 ± 82.76	289.34 ± 100.55	138.24 ± 110.89	0.001
2 (caffeine)	151.20 ± 64.03	231.05 ± 49.82	79.84 ± 56.86	0.001
3 (fluoride)	146.29 ± 69.26	291.82 ± 94.51	145.53 ± 84.43	0.001
4 (distilled water)	149.98 ± 64.42	209.15 ± 57.24	59.16 ± 53.38	0.001
	0.996	0.004	0.003	

Diff 2 = remineralization–demineralization; SD: standard deviation.

**Table 3:** Comparison of microhardness values in pairwise groups.

Group	Theobromine	Caffeine	Fluoride	Distilled water
Theobromine	—	0.035	0.780	0.005
Caffeine	0.035	—	0.017	0.460
Fluoride	0.780	0.017	—	0.002
Distilled water	0.005	0.460	0.002	—

## Data Availability

All the data generated or analyzed during this study are included in this published article, and the datasets used to support the findings of this study are available from the corresponding author upon request.
